# Government Environmental Governance and Enterprise Coordinated Green Development under the Goal of “Double Carbon”

This article has been retracted.

**DOI:** 10.1155/2022/6605935

**Published:** 2022-06-21

**Authors:** Fang Liu, Jingjun Jiang, Shuwen Zhang

**Affiliations:** ^1^School of Economics, Zhongnan University of Economics and Law, Wuhan, Hubei 430000, China; ^2^Business School, Henan Normal University, Xinxiang 453000, China; ^3^Law School & Intellectual Property School, Jinan University, Guangzhou 510632, China

## Abstract

China's 13th five-year plan puts forward the development concept of “green development” and takes the construction of green financial system as the development strategy, which shows that the concept of environmental governance and green development is becoming more and more important for national economic development. It is a major strategic task for China to build an environmental governance system dominated by the government and dominated by enterprises and implement the main responsibility of enterprise environmental governance. At present, the environmental supervision of local governments needs to be improved urgently. It is necessary to strengthen the production regulation of enterprises and promote the emission of “three wastes” up to the standard based on the principle of “polluter pays.” The green development of enterprises is not only conducive to the improvement of their own “three effects” and corporate image but also has the external spillover effect of giants and is conducive to the construction of ecological civilization. Therefore, this study will focus on the collaborative governance in the field of environment, explore the ideal collaborative governance framework in the process of environmental collaborative governance, as well as the difficulties and optimization paths of collaboration, and put forward corresponding suggestions for the current environmental governance.

## 1. Introduction

The report of the 19th National Congress of the Communist Party of China regards pollution prevention and control as one of the three key battles to win the decisive victory in building a well-off society in an all-round way and puts forward the construction of an environmental governance system dominated by the government and dominated by enterprises, to implement the major strategic task of the main responsibility of enterprise environmental governance [1]. Polluters are the main body responsible for pollution control. Strengthening their environmental protection responsibility will help to improve environmental quality and promote the formation of a standardized and fair market competition environment. The transition of China's economy from high-speed growth to high-quality growth is not only due to the transformation of demand by the dynamic mechanism of economic growth but also forced by the actual situation of bearing pressure on China's resources and environment. In the past high-speed economic growth stage, it was mainly based on the development of heavy industry economy, which inevitably caused serious pollution problems. This shows that the source of environmental pollution is industrial enterprises, especially those in heavy pollution industries. Therefore, if we can effectively control the pollution emission of heavy polluting enterprises, it will certainly bring China's environmental governance to a higher level [2].

Based on the urgent need to improve China's ecological environment, the growing desire of the people to “look forward to environmental protection” and “seek ecology,” the increasing pressure of enterprise transformation and upgrading, and the urgent need for correct guidance of the development concept and performance view of some local leading cadres, how to test the effectiveness of local environmental governance construction and development and optimize the coordination path according to the problems, shortcomings, and difficulties in the current local governance practice improving the governance system is in line with the practical needs of China's adherence to the green development strategy and will play a key role in China's practice of the concept of green development [3].

## 2. Concept Definition and Theoretical Basis

### 2.1. Concept Definition

#### 2.1.1. Enterprise Green Development Model

As a profit-making organization, enterprises naturally have the pursuit of profits. The rapid development of enterprises has created conditions for the pursuit of profits. Compared with the traditional development model, the green development of enterprises is a development model different from the previous development model with green as the core, which is a sustainable enterprise development model. Green development of enterprises is a new green-oriented development model. This development model meets the standards of resource conservation and ecological civilization and belongs to an important part of the construction of ecological civilization. Under the background of vigorously promoting the construction of ecological civilization, the green development of enterprises is facing unprecedented opportunities and challenges. The green development of enterprises belongs to the category of green development, but the main body is enterprises. Therefore, it has the general characteristics of green development and has the characteristics of maintaining the unique green development of enterprises [4].

*(1) Strategic and Long Term*. Enterprise green development belongs to a new enterprise development model, which is different from the traditional non-green development model. This development model pursues the overall strategic green development of the enterprise. Enterprise green development is not only the need of a certain department or stage of the enterprise but also the development model of the enterprise as a whole involving all departments of the enterprise and includes the development model of each stage of enterprise development. Therefore, it has strong integrity and strategy. At the same time, we should make strategic arrangements and realize the needs of green development. At the same time, the green development strategy of enterprises is not the development needed for a while, but the development model that needs to be adhered to for a long time. Enterprise green development belongs to a development model that can bring long-term benefits, and this benefit can only be obtained in the process of long-term persistence. Therefore, whether considering the current interests or long-term strategic thinking, enterprises need to adhere to the development model of green development for a long time [5].

*(2) Comprehensive and Phased*. In addition to long-term planning, the green development of enterprises also needs richer connotation and comprehensive consideration and thinking. The green development of enterprises needs comprehensive design and planning, and the green development strategy and planning of enterprises must be well designed. Enterprise green development also needs to redesign the system and mechanism design of enterprise green development [6]. The system suitable for green development is to arrange the organization and distribution of rights and responsibilities of enterprise green development; the mechanism suitable for enterprise green development is to consider the institutional method of enterprise green development [7]. Enterprise green development also needs to pay attention to the establishment of enterprise green development consciousness, to create a good enterprise green development culture [8]. Therefore, the green development of enterprises needs comprehensive consideration and planning. At the same time, the green development of enterprises has a long-term development stage. Different enterprises are in different green development environments at different development stages and have different needs for green development. Moreover, the same enterprise has different needs at different stages of development [9]. Therefore, the green development of different enterprises and different development stages has different development modes, and the green development of enterprises has the characteristics of stages [10].

*(3) Innovation and Difference*. Enterprise green development is a concept with rich connotation, and it is a concept of continuous innovation. The green development of enterprises is put forward on the basis of the deterioration of resource problems and environmental problems [11]. The main purpose is to promote the green development of the whole society through the green development of enterprises. The initial green development of enterprises is more from the perspective of development consciousness and development concept [12]. The real green practice is still limited, mainly to deal with the internal sustainable development and efficiency of enterprises. Later, with the gradual deepening of the concept of green development, the connotation of enterprise green development gradually expanded [13]. In addition to meeting the needs of the enterprise itself, it also needs to further meet the needs of the enterprise's external environment and produce positive external effects. Therefore, the connotation and extension of enterprise green development are expanding and innovating. As environmental protection has become a global issue, different countries and regions are bound to encounter this problem, which will put forward more or less requirements for the green development of enterprises. However, due to the different national conditions and practical needs, the green development strategies of different countries and regions are very different [14].

#### 2.1.2. Multicenter Collaborative Governance

Both “collaborative governance” and “polycentric governance” are facing the realistic changes that social governance urgently needs the wider participation of public or private stakeholders and form a multilateral decision-making process aimed at directly formulating or implementing governance policies and management plans. To form such a consensus and efficient governance system, whether it is “collaborative governance” or “multicenter governance,” we should make an effective balance between risks and benefits, ensure positive interdependence among stakeholders, and make the cooperation process fair, inclusive, and complementary.

However, it is obvious that the simple and blind pursuit of “multicenter” will undoubtedly lead to the defects of coordination and complementarity in the process of cooperation and make governance become the surface form of “metaphysics,” which can not go deep into the root causes to solve the problems of social governance. Similarly, relying solely on “synergy” to solve governance problems will also lead to the compromise of all actors in order to achieve a unified goal, and the interests of all parties cannot be guaranteed; in particular, the needs of vulnerable subjects will be excessively ignored. To make multicenters play an effective role in the collaborative process, we should not only avoid the split of all parties but also avoid compromise. Therefore, we integrate the multicenter theory and synergetics into the field of governance and establish a collaborative governance model with the participation of multiple subjects, so that multiple centers can effectively perform their respective duties, cooperate with each other, and give greater play to the collaborative effect.

### 2.2. Theoretical Basis

#### 2.2.1. Collaborative Governance Theory

Collaborative governance means that under the open framework composed of various power subjects in social public life, through administrative, legal, technical, public opinion, and other means, the originally chaotic elements coordinate and interact with each other to form an orderly collaborative system, so as to effectively manage public affairs and finally achieve the purpose of safeguarding public interests. According to the theory of collaborative governance, the government, enterprises, and people can all be participants in public affairs, and the common interest has become the key point affecting the decision-making behavior of different participants. Whether the participants can intervene and express depends on their “ability to raise and solve problems” [15].

First is the overall goal of overall coordination. It can not only meet the requirements of multi interests but also mobilize the enthusiasm of multi-governance subjects to participate in governance. Second, the collaborative governance system is an open system [16]. In this system, the subjects participating in governance have the characteristics of diversity, and the diversity of participants also requires the openness of the governance system [17]. Only in an open environment can all market players, nongovernmental organizations, and the public except the government have the opportunity to participate in governance. Subjects can achieve governance objectives through equal consultation, negotiation, and cooperative action and finally maximize local and overall interests. Third, the process of collaborative governance is a dynamic process [18]. Due to the uncertainty of the environment, the relationship between local environmental cooperation and governance subjects, the objectives of different stages, governance objects, and the organizational framework, cooperation rules, and resource exchange in the governance process are dynamic. Fourth, the boundary of collaborative governance is relatively vague. In the process of collaborative governance, under the action of synergy, the boundary of the original subsystem becomes more blurred due to the close relationship between subsystems. It is mainly reflected in the fuzzy boundary of the governance scope of public affairs and the fuzzy boundary between the governance subjects [19]. The fuzzy boundary is conducive to the better governance effect of collaborative governance. In addition, the biggest feature of collaborative governance is the diversification of its governance subjects as shown in Figure 1. Under collaborative governance, the leading role of the government and the participation of multiple governance subjects in various social departments are the manifestations of the participation of multiple governance subjects as shown in Figure 2 [20].

#### 2.2.2. Stakeholder Theory

Potential conflicts of interest between managers and stakeholders or between stakeholders also blur their definitions and roles. Based on the characteristics of different attributes, stakeholders can be divided into deterministic stakeholders, expected stakeholders, and potential stakeholders. The priority of deterministic stakeholders to the three key attributes is power, legitimacy, and urgency. It is proposed that more consideration needs to be given to primary and secondary stakeholders in order to effectively allocate and manage scarce resources. However, key stakeholders are more important to the survival and well-being of enterprises. Therefore, some scholars emphasize that there is a considerable gap between the interests of stakeholders understood by a key organization and the interests perceived by stakeholders themselves. Some scholars believe that this dichotomy may lead to unexpected resistance among stakeholders in the process of implementing management decisions. Therefore, the concept of “stakeholder diversity” is proposed, emphasizing that management must recognize that stakeholders are part of the network rather than a “binary image.”

Stakeholder theory was initially applied in the field of economic management. With the development of relevant research, this theory has gradually developed in the field of public management and has been widely used in the research of government, citizens, and nonprofit organizations in the third sector. In the field of environment, all citizens live in it. As the direct bearers of ecological change, they have the most say in ecological governance in the face of the infringement brought by ecological damage. Therefore, stakeholder theory is an important theoretical basis for citizens to participate in ecological governance. To realize the long-term development of the country, the government's ecological governance must include multiple stakeholders in the ecological governance, achieve the consistency of governance objectives through consultation and cooperation, and finally achieve governance results.

#### 2.2.3. Environmental Kuznets Curve Theory

The environmental Kuznets curve shows the impact of economic development on the degree of environmental pollution through the evolution simulation between per capita income and environmental pollution indicators; that is, in the process of economic development, the environmental situation deteriorates first and then improves gradually. The theoretical explanation of this relationship mainly focuses on three aspects: economic scale effect and structure effect, the relationship between the demand for environmental services and income, and the government's policies and regulations on environmental pollution.

After the environmental Kuznets curve hypothesis was obtained, many experts made research using the pollution data in different regions and found that the curve hypothesis was valid in most cases. In the initial stage of economic development, the per capita income is low, mainly due to the negative effects of social scale expansion and social structure changes. With the increase in per capita income, environmental pollution will inevitably fall into an irreversible situation. However, when the per capita income reaches a high level, technological change and social structure change will have a positive effect on the environment. The per capita income will increase, but the environment will not deteriorate and tend to improve. In addition, in the actual process, because the degree of environmental regulation is not necessarily “inverted U,” there are three other similar curves. After the environmental Kuznets curve was proposed, a large number of scholars calculated the specific value of the inflection point of the environmental Kuznets curve through the analysis of the data database of each region and country, which can be obtained through verification. They believe that this is the inevitable result of environmental pollution and social development. If a government is laissez faire to the environment, those countries that have gone through the development model of pollution before treatment are the lessons of developing countries as shown in Figure 3.

## 3. Current Situation of Environmental Collaborative Governance in China

### 3.1. The Differences in the Forms of Environmental Regulation Lead to the Heterogeneity of Green Development of Enterprises

Enterprise green innovation can include green management innovation, green process innovation, green product innovation, and green technology innovation. However, due to the consideration of quantifiable form and the impact on the effect of environmental pollution control, this study only selects the green technology innovation of listed companies in heavy pollution industry as the research object. The final empirical results show that both command-based and market-based environmental regulations have a significant role in promoting enterprise green innovation. Among them, market-based environmental regulation is selective in a more flexible way, and its role in enterprise green innovation is stronger than command-based regulation, while public participation in environmental regulation has no significant role in green innovation due to less administrative binding force and imperfect system construction. In addition, the moderation of environmental regulation intensity has a threshold effect on green innovation, but it only exists under the means of imperative environmental regulation. There is an inverted “U” structural relationship between them. Moderate imperative regulation can promote the green innovation of enterprises to reach the optimal value; there is only one-way linear relationship between market-oriented and public participation environment. In addition, giving executives different compensation and equity incentives plays a significant positive role in promoting the output of green innovation under the role of regulation, but relatively low equity incentives and higher salary incentives are more conducive to the green innovation of enterprises. The above results show that environmental regulation is an important means to promote the output of green innovation of enterprises, especially the market-based regulation means. To solve the environmental pollution from the root, we should take the market-based regulation means as the leading, supplemented by the command-based regulation means with appropriate intensity, and gradually improve the construction of public participation regulation tools. In addition, when strengthening the output of green innovation within enterprises, we can consider supplementing the lack of external regulation through the management incentive system of low equity and high salary.

### 3.2. Under Environmental Regulation, Enterprises Should Pay Attention to the Change in Concept, from Passive Emission Reduction to Active Green Innovation

Since the 1990s, a “green revolution” has sprung up all over the world. The issue of environment and development has become the center of a new round of multilateral trade negotiations, namely the “green round.” As the WTO allows member states to take corresponding measures to strengthen environmental protection, green barriers will inevitably exist and become the most important “disguised trade barriers.” To follow these green trade rules, break through green barriers, and avoid trade sanctions, enterprises must implement green brand strategy to achieve rapid and healthy development.

The construction of ecological civilization has penetrated into people's daily life. It can be verified from the pilot of waste classification in Shanghai. On the one hand, it shows that the government has strengthened the governance of ecological environment; on the other hand, it shows that the concept of environmental protection has been rooted in every public heart. The enhancement of public awareness of environmental protection will certainly guide the upgrading of consumers' consumption ideas, and green environmental protection and clean energy products will be highly respected. If enterprises can convey the concept of proactive environmental governance to the outside world, they will be recognized by more consumers and investors and increase the competitiveness and economic value of enterprises.

### 3.3. Preliminary Practice of Enterprise Green Strategy

When seeking development, enterprises should adhere to the requirements of sustainable development and organically combine the concept of green environmental protection with production activities, so that their own interests and the cause of green environmental protection can be win-win, and economic development and ecological development can be coordinated, to finally achieve the perfect consistency of social interests, collective interests, enterprise interests, and ecological interests and realize real sustainable development. To achieve consistency, our enterprises are required to realize their own interests while taking the protection of the ecological environment as the basis and always bear in mind that social interests, collective interests, and ecological interests are above everything. It is the premise for enterprises to realize their own interests and develop. Enterprises can carry out normal production and life activities only on the premise of not violating social interests, collective interests, and ecological interests to truly realize the long-term development of the enterprise itself. Enterprise green culture management requires enterprises to consider the importance of natural resources in the process of production and sales. We must stop the production activities at the cost of polluting the environment. Our entrepreneurs are required to have the awareness of green environmental protection and really care about the long-term development of the enterprise, not just the short-term development. When managing, our entrepreneurs should really achieve the management decision of sustainable development, the management awareness of green culture of environmental protection, and the strategic planning of long-term development of the enterprise. A key point is firmly grasped—the cultivation and application of green management ideology, change passivity into initiative, actively control the environmental protection cost in the production cost, refine the enterprise green culture management, and do not be eager for quick success and instant benefit, only pursue short-term immediate interests, and lose the opportunity to obtain greater long-term interests. What entrepreneurs should think about is how to realize the benign and sustainable development of enterprises themselves? If enterprises want to realize standardization in production activities, they need to have a set of perfect management rules, and the rules will form a system when they are implemented. If entrepreneurs want their enterprises to achieve sound and sustainable development, they must have a set of sound rules. Only the awareness of green culture management is not enough. They must be applied to the scarf of action in order to play a role.

### 3.4. Current Situation of Environmental Governance

The environmental data of Shanxi Province are taken as an example.

The number of environmental protection departments and staff is increasing. The number of environmental protection departments and the number of personnel in the environmental protection system can reflect a region's attention to environmental governance from one side. To strengthen the task of environmental governance in Shanxi, environmental degradation is improved and protection management is promoted, and the number of protection institutions above the county level in Shanxi Province has gradually increased since 2006. By 2016, the number of protection departments above the county level in Shanxi Province had reached 792; the number of protection system personnel in the province is 13165 as shown in Figure 4.

The overall investment in emission control projects is increasing. From 2006 to 2017, the investment in the completion of emission control projects in Shanxi Province showed an increasing trend. In 2006, the investment in emission control in Shanxi Province was 33.54 billion yuan, and it then gradually increased. By 2016, the investment in industrial emission and the number of projects reached a record 52.58 billion yuan, ranking first in previous years, but the investment in 2017 decreased slightly as shown in Figure 5.

From 2000 to 2017, the total amount of major emissions in Shanxi Province was gradually reduced, and the emission standard rate of major emissions was rising. From 2006 to 2017, the comprehensive utilization capacity of garbage and the treatment capacity of domestic garbage in Shanxi Province were also improved with the increase in environmental governance. All these show that in recent years, the intensity of environmental governance in Shanxi Province has indeed shown an upward trend as shown in Figure 6.

From the perspective of industrial wastewater discharge, generally, the wastewater discharge was high from 2000 to 2014. Since 2014, wastewater discharge has decreased significantly year by year. In particular, after 2016, the discharge of industrial wastewater has reached a new low. It proves that the current environmental protection work of industrial wastewater discharge cover is done well as shown in Figure 7.

Between 2000 and 2017, sulfur dioxide emissions are divided by 2011. Until 2011, sulfur dioxide emissions have been high and occasionally decreased in individual years, but the overall trend is upward, but after 2011 sulfur dioxide emissions continued to decline, especially after 2015, with a rapid decline of nearly 400000 tons of sulfur dioxide emissions in one year as shown in Figure 8.

From 2006 to 2017, the harmless treatment rate of domestic waste in Shanxi Province has always maintained an upward state. It can be seen that the harmless treatment of domestic waste in China is developing and progressing as a whole.

## 4. Suggestions on Strengthening Coordinated Environmental Governance

### 4.1. Maintain Appropriate Mandatory Environmental Regulation and Gradually Improve the Construction of Market-Oriented and Public Participation Environmental Regulation Systems

Because the mandatory environmental regulation emphasizes the punishment of environmental governance, the moderate intensity of environmental regulation has a positive role in promoting the green innovation of enterprises. However, when the regulation is too strict and the governance cost is too high, it may lead to the negative governance attitude of enterprises, but it violates the original intention of the mandatory environmental regulation system. In the future regulation construction, we should provide reasonable guarantee for the channel of public advice and suggestions, to urge enterprises to take the initiative in environmental construction under the pressure of public opinion supervision. Perfect environmental regulation plays a positive role in promoting sustainable economic development. According to relevant research, effective and standardized environmental regulation will have a positive impact on enterprise technological innovation. Perfect environmental protection incentive mechanism can encourage industrial enterprises to innovate. A green technology innovation system is established with enterprises as units and industrial enterprises are urged to invest in technological innovation, so that industrial enterprises can obtain competitive advantages and occupy the commanding height of competition. Adhering to innovation leading and deeply implementing the innovation-driven development strategy, the government and enterprises should take scientific and technological innovation as the first driving force to lead industrial development. By strengthening environmental regulation, enterprise technological innovation is stimulated and production efficiency is improved, to walk in the front of the production industry. At the same time, in the environment of industrial structure reform and transformation, environmental regulation tools must also be improved. In addition to strengthening command-based environmental regulation means, we should also combine market-oriented environmental regulation and administrative environmental regulation, such as closely combining environmental tax, emission tax, and emission trading system, and adopt diversified environmental regulation tools to improve the status of laws and regulations in industrial production.

### 4.2. Strengthen the Information Transmission Function of Media Environment and Realize Multi-Agent Collaborative Governance

The increase in media attention to enterprises can not only urge enterprises to improve their external environmental performance to meet the regulatory requirements but also promote enterprises to actively carry out green innovation and cut off the source of environmental pollution from the root. The positive regulatory effect of media attention on environmental regulation and enterprise economic performance shows that media attention expands the “win-win” effect of simultaneous growth of environmental and economic benefits. Therefore, in the future environmental construction, the government and the public should pay more attention to the transmission function of media to environmental information and reputation transmission mechanism, give full play to the information media role of media, and realize the formal governance model of multi-agent participation in environmental governance. The government's environmental regulation is strengthened and a sound environmental information disclosure system is established. The government plays a leading role in environmental governance, but due to the inconsistency of interest objectives between the central and local governments, local governments may choose to ignore environmental pollution and give priority to the development of regional economy. Information asymmetry also provides a possible space for local governments to weaken the implementation of environmental policies. Therefore, it is necessary to establish a sound local government information disclosure system and earnestly implement the inclusion of environmental performance into the performance evaluation of officials, to effectively supervise the implementation of local government environmental policies and strengthen the government's environmental regulation. At the same time, the central government can also establish cooperative relations with environmental protection social organizations, give play to the effective supervision role of environmental protection social organizations, and use various pressures to ensure the effective implementation of environmental policies of local governments.

### 4.3. Strengthen Government Guidance

At this stage, China attaches great importance to environmental protection, and green development has become an inevitable requirement for building a modern economic system. Relevant systems are reformed, relevant regulations are improved, and high-quality development and environmental protection are coordinated and promoted. In the face of the increasing shortage of resources and the aggravation of environmental pollution, the environmental protection department should formulate industrial plans to implement environmental improvement. It cannot simply and roughly achieve one size fits all. It should correctly guide industrial enterprises to develop in the direction of resource-saving and environment-friendly. The coordinated development of modern environmental policy is based on environment and economy. Promoting the coordinated development of economy and environment is not only related to the effective implementation of regulatory policy but also related to the implementation efficiency of laws and policies. Enhancing the effect of environmental regulation is very important for industrial green development. Relevant functional departments should strengthen the compulsion of environmental regulation, ensure the implementation of environmental regulation from formulation to implementation, supervise and urge the implementation of the work of departments at all levels in the process of environmental regulation, guide and supervise the behavior of industrial enterprises, and give certain punishment measures in case of noncompliance. In terms of specific measures, first, environmental governance training is strengthened. We should not only carry out environmental governance training for enterprise leaders but also carry out in-depth training on environmental protection laws and regulations for local enterprise managers and employees, to enable the people to establish environmental protection awareness and green production awareness and urge enterprises to take the initiative to bear social responsibility. Secondly, local governments can innovate guidance methods and introduce enterprises to participate in environmental governance. Local governments estimate the participation of enterprises in environmental protection actions by combining administrative guidance, and attention should be paid to the smoothness of channels in the process of strengthening market supervision, to increase the enthusiasm of enterprises to participate in environmental governance. Finally, enterprises link interests with social responsibility. Local government departments should support and guide enterprises to comprehensively carry out environmental labeling product certification, establish a corporate image, and link corporate interests with social responsibility, to improve the motivation of enterprises to participate in environmental protection governance.

### 4.4. Enterprises Should Change Their Development Ideas and Promote the Transformation and Upgrading of Enterprises

With the development of the times and the increasing requirements of environmental protection, the traditional development concept needs to be updated. At present, China has entered the new normal period of economy. Adjustment, transformation, and upgrading have become the keywords of this era. Industrial transformation and upgrading are an important issue in this period. If enterprises want to adjust their traditional development concept, they cannot take economic interests as a single goal, nor can they take the environment as the price of economic development. On the one hand, enterprises can develop their low-end industrial chain into high-end industrial chain. Enterprises can extend their own industrial chain and promote the development of the whole industrial chain in the direction of low energy consumption and low pollution. The investment of enterprises cannot be limited to the production range of the original enterprise, but also invest in emerging investment fields and expand their own investment fields. It not only promotes the improvement of the overall income of the enterprise but also improves the anti-risk ability of the enterprise. On the other hand, industrial enterprises can change the traditional process, upgrade the process flow and production equipment, reduce pollution emissions, adopt more advanced energy-saving technology, improve the added value of products, and promote the transformation and upgrading of industrial enterprises and realize green development in these ways. The subjective initiative of green transformation of enterprises is stimulated and actively guided to carry out green production. Enterprises are the main source of pollutant emissions. How to strengthen and guide the green transformation of enterprises should be a key issue in environmental governance. Government departments should strengthen the incentive of enterprises' environmental protection behavior, help enterprises realize green production, and provide financial subsidies and more social resources to enterprises that realize green transformation, to effectively stimulate the subjective initiative of enterprises' green transformation. In addition, environmental protection social organizations can also establish cooperative relations with enterprises, use their professional advantages to provide support for the green transformation of enterprises, and use their advantageous position in the public to publicize the products of green transformation enterprises, guide consumers to buy green products, and improve the competitiveness of enterprises, to stimulate enterprises to have more power of green transformation.

(1) Strengthen the Cultivation and Accumulation of Human Capital. Human resources are the internal driving force for the survival and development of modern enterprises and an important basis for the sustainable development of enterprises. Now, all provinces have vigorously implemented the talent development strategy, seized talent resources, and accelerated the establishment and improvement of the innovation system. While cultivating their core innovation strength, enterprises should also establish their own talent introduction policies and vigorously introduce innovative talents from various universities and research institutes. We should cultivate our own talents in some key fields and links related to enterprise development. (2) Enterprises should vigorously promote the transformation of scientific and technological achievements, protect the legitimate rights and interests of legitimate owners, establish a long-term incentive mechanism, and promote enterprises' continuous innovation. (3) We should establish an innovation atmosphere for enterprises and encourage innovation. Innovation should not only stay at the slogan level of the enterprise but also should become the consensus spirit of the enterprise. Innovation should become the core concept and core culture of the enterprise and go deep into everyone's heart.

### 4.5. Enterprises Should Improve Their Sense of Social Responsibility

Corporate responsibility cannot be missing in any period. Industrial enterprises bear great responsibility in the process of environmental regulation. The fulfillment of social responsibility by industrial enterprises is the key to ensure the normal operation of the economic market and the sustainable green development of enterprise activities. Enterprises should not only improve the quality of products but also establish a good brand image. First of all, enterprises should establish a perfect internal supervision mechanism in production activities to prevent pollution loopholes. Enterprises should not only control the environmental protection standards of production methods or raw materials at the source of production but also ensure that products meet the standards, make more use of clean technology, and improve the green quality of products. Secondly, industrial enterprises should actively respond to the government's environmental protection policies, such as actively cooperating with the government's legal implementation, actively cooperating with other enterprises, and demanding themselves with higher environmental regulation standards in the process. In the process of development, heavily polluting enterprises will inevitably have a negative impact on their corporate image, and enterprises that make outstanding contributions to environmental protection can win the favor of the market. Enterprises can improve their sense of responsibility from the aspects of product concept, sales mode, and production capacity, to realize the unified development of enterprise economic growth, social environment, and natural environment. The future of society is also the future of enterprises. The better the corporate social responsibility is, the more conducive to the implementation of environmental regulation and the green development of enterprises.

## 5. Conclusion

It is undeniable that in the process of environmental governance improvement, the coordination of multiple governance subjects and social groups is essentially important. The restriction and running in of the relationship between the main bodies such as organizations, citizens, and government are a problem that needs long-term attention. Straightening out the division of labor and relations among various subjects in the process of collaborative governance is not an overnight process. However, we should also note that collaborative governance of the environment is an inevitable choice to meet the social needs and respond to the needs of citizens. Collaborative governance is the result of the continuous socialization of public management functions in contemporary society, which means not only the continuous decentralization of governance authority but also the complete transformation of the government's governance concept and economic development mode. This means that in the process of traditional public management, the “top-down” management mode of society and market marginalization and pure government as the center is changing into a new governance model, which means that the original concept of seeking development at the expense of the environment will also be completely changed under the new environmental governance model; that is, the market, society, and citizens are the main participants and take a strong government as the core and leadership. Coordination and cooperation are maintained with each other and worked together to maximize the benefits of environmental protection affairs and improve the quality and efficiency of public environmental services. Therefore, overcoming the obstacles in the process of collaborative environmental governance requires the cooperation of various principles, systems, and process management, so that different stakeholders can establish a relationship of mutual trust, mutual reliance, and mutual understanding under their governance capabilities.

## Figures and Tables

**Figure 1:** System framework of China's environmental collaborative governance.

**Figure 2:** Logic of environmental governance in China.

**Figure 3:** Environmental Kuznets curve.

**Figure 4:** Number of full-time personnel in the environmental department.

**Figure 5:** Total investment in environmental pollution control in Shanxi Province.

**Figure 6:** Industrial wastewater discharge (10000 tons).

**Figure 7:** Sulfur dioxide emission (10000 tons).

**Figure 8:** Harmless treatment rate of domestic waste.

## Data Availability

The labeled data set used to support the findings of this study is available from the corresponding author upon request.
